# Influence of Classical Massage on Biochemical Markers of Oxidative Stress in Humans: Pilot Study

**DOI:** 10.1155/2021/6647250

**Published:** 2021-12-10

**Authors:** Zofia Skubisz, Daria Kupczyk, Aleksander Goch, Marcin Siedlaczek, Łukasz Sielski, Bartłomiej Niespodziński, Emilia Mikołajewska, Mariusz Zasada, Beata Augustyńska

**Affiliations:** ^1^Institute of Physical Education, Kazimierz Wielki University in Bydgoszcz, Poland; ^2^Department of Medical Biology and Biochemistry, Ludwik Rydygier Collegium Medicum in Bydgoszcz, Nicolaus Copernicus University, Toruń, Poland; ^3^Department of Physiotherapy, Ludwik Rydygier Collegium Medicum in Bydgoszcz, Nicolaus Copernicus University in Toruń, Poland; ^4^Ludwik Warmiński Municipal Hospital in Bydgoszcz, Poland

## Abstract

Classical massage is one of the most popular forms of conservative treatment in various diseases. Despite the wide scope of research, the mechanisms of massage are not fully known and understood. Apart from the well-described effects on individual body systems, there are few scientific reports on the effects of massage on the human body at the subcellular level. The study was designed to assess changes in oxidative stress parameters in healthy volunteers after a single session of classical massage. 29 healthy volunteers aged 22.24 ± 3.64 participated in the study. Before and 30 minutes after the massage procedures, blood samples were taken by experienced personnel. Biochemical markers of oxidative homeostasis were assessed with highly specific methods for each parameter: oxidase ceruloplasmin, glutathione, malondialdehyde, glutathione peroxidase, glutathione S-transferase, and superoxide dismutase. The study demonstrates that massage therapy caused statistically significant decrease in the concentration of glutathione peroxidase (red blood cells) and increase in the level of glutathione peroxidase (plasma), superoxide dismutase, and malondialdehyde. In contrast, statistically significant changes in the hematocrit, glutathione, NO_2-_/NO_3-_, and oxidase ceruloplasmin were not observed. The results show that complex influence of classical massage therapy on human organism may be reflected in parameters of the oxidative stress. To understand this mechanism clearly, further research is needed.

## 1. Introduction

Oxygen is involved in many metabolic processes. It plays a role of an oxidant. During the reaction with organic compounds, it collects electrons and undergoes a process of reduction. When reduction process of oxygen molecules is incomplete, reactive oxygen species (ROS) may be formed [1–3]. Reactive oxygen species include neutral molecules or ions and oxygen free radicals, i.e., atoms or molecules that have at least one or more unpaired electrons [4, 5]. Among ROS, the following should be named: alkoxy radical RO, radical ROO peroxide, singlet oxygen O_2_, ozone O_3_, hydrogen peroxide H_2_O_2_, superoxide anion O_2-_, and hydroxyl radical OH [6]. ROS easily react with cell elements which may lead to changes in the cell structure and numerous damages. ROS play an important role in maintaining homeostasis: they influence signaling cells or relay cells, providing proper cell metabolism [4, 7]. ROS also participate in functioning of the immune system, excretion of hormones, contraction of muscles, and muscle tone regulation.

There are defense mechanisms within the human organism which guard against ROS activity [4], including, e.g., antioxidative enzymes: superoxide dismutase (SOD-1), catalase (CAT), glutathione peroxidase (GPx), glutathione reductase (GR), glutathione S-transferase (GST), and glutathione (GSH), vitamin E, vitamin C, bilirubin, ceruloplasmin (CP), uric acid, ferritin, and transferrin. Extensive production of ROS and inefficient action of the antioxidant defense mechanisms cause negative results. Oxidation reaction may be unbalanced which leads to a phenomenon called oxidative stress [8, 9]. The human body may be exposed to numerous environmental factors, such as unhealthy food, alcohol, cigarette smoke, medications, stimulants, air pollution, and pathogenic microorganisms, which may provoke generation of various oxygen forms in the organism [10]. Every prohealth initiative such as physical activity, optimal diet, and physiotherapy may decrease the risk of free radical-related diseases. Numerous studies show the influence of physical activity on oxidative stress parameters but there is a lack of research into the effect of therapeutic massage on oxidative stress parameters [11–13].

Massage therapy still remains a popular and natural way of treatment, constituting part of health prevention. During years of evolution of soft tissue therapy, a lot of different types of massage were developed all over the world. Classical massage, also called Swedish massage, is very a complex and standardized activity which consists in using successive techniques of effleurage, friction, petrissage, tapotement, rolling, shaking, and vibration [14].

Depending on the technique, massage may energize or relax tissues and systems. It acts both locally and, through the central nervous system, globally. Classical massage has an effect on functioning of the human body on various levels, from cells to whole systems, including nervous, circulatory, pulmonary, digestive, urinary, and endocrine system [15, 16]. Thus, the influence of massage on the body can be described as complex and diverse. Literature also frequently describes a decrease in cortisol levels, changes in blood parameters, or an increase in dopamine levels, which has a positive effect on the patient's well-being [16, 17]. This is explained by the fact that the mechanical stimulus changes the activity of the vagus nerve, putting the patient in a parasympathetic state leading to a regeneration reaction. An increase in the presence of NK cells as well as CD4 is also observed. Similarly, the immunity is positively influenced by chromogranin A which was described by Noto et al. [18]. Hypothesis stating that such complex influence may be reflected in parameters of the oxidative stress can be true. Massage as a mechanical stimulus can potentially cause microtrauma in connective tissue, which may correspond to some of the effects of physical activity and, as a consequence, trigger an antioxidant reaction.

Until now, the evidence for such impact is limited and more concentrated on physical activity or combination of physical activity and massage [19, 20]. In the available literature, no publications that deal exclusively with the topic of the influence of massage on the antioxidative response were found. Therefore, the given study is aimed at assessing the human early antioxidative response to the single classical massage session [11, 19].

## 2. Material and Methods

### 2.1. Material

The study group consisted of 29 healthy people (15 females and 14 males) mean age 22.24 ± 3.64 years, with no health conditions (fever, contagious diseases, blood clots, pregnancy, kidney and liver conditions, cancer, inflammations, and hypertension were excluded as a contraindication during general medical examination). The assessed group did not have regular massages previously. Participants were not practicing sport professionally and have no regular medications, addictions, obesity (BMI between 19 and 23), or diabetes. Every person was fasted till the last blood sample collection.

This study was conducted in accordance with the Declaration of Helsinki and approved by the local institutional review board. Freely given written informed consent was obtained from every patient prior to the study.

### 2.2. Methods

Participants were treated using classical massage therapy in the Department of Physiotherapy, Ludwik Rydygier Collegium Medicum in Bydgoszcz, Poland. Every patient had one session of the massage for at least 30 minutes. The classic massage covered the dorsal part of the torso, including the spinal and dorsal area (lateral part of abdominal oblique muscles, trapezius, rhomboids, latissimus dorsi, and erectors of the spine). The procedure was carried out under repeatable and unified conditions for the whole group, by one experienced physiotherapist with intermediate intensity, without crossing pain barrier. The massage consisted in the use of successive techniques of effleurage, friction, petrissage, tapotement, rolling, shaking, and vibration, in accordance with the standard of their performance. Blood samples were collected twice: before massage and after the massage.

In the experiment, activity of following biochemical markers of oxidative homeostasis was assessed: oxidase ceruloplasmin (CP), glutathione (GSH), malondialdehyde (MDA), glutathione peroxidase (GPx), glutathione S-transferase (GST), and superoxide dismutase (SOD-1).

The material for analysis was venous blood collected in an amount of approx. 8 ml of the antecubital vein into lithium heparin tubes and tubes without anticoagulant. First blood samples were collected in the morning from 8.00 to 9.00 before massage, and second were 30 minutes after procedure. Then, collected material was transported to laboratory. Tests were carried out on the same day in the Department of Biochemistry of Nicolaus Copernicus University Collegium Medicum in Bydgoszcz, within one hour of material collection. From the blood drawn into tubes without anticoagulant (approx. 3 ml) serum was obtained by centrifugation of the material over 5 min at 5000 × g; then it was transferred to Eppendorf tubes and frozen at -80°C. The prepared serum was stored to determine the activity of the oxidase ceruloplasmin (CP). Before preparing the hemolysate, 500 *μ*l blood was collected to determine the levels of glutathione (GSH) in the erythrocytes, and the remaining aliquot of blood (approx. 5 ml) was centrifuged to obtain plasma, wherein the concentration of nitrate/nitrite was determined. The remaining cells were used for the preparation of the hemolysate, wherein the dialdehyde malonic concentration (MDA) and the activity of the enzymes glutathione peroxidase (cGPx), glutathione S-transferase (GST), and superoxide dismutase (SOD-1) were determined.

The concentration of reduced glutathione (GSH) was assayed using the Beutler method [21]. The principle of this method is based on the reaction of reduction of the disulfide compound—dithio-bis-2-nitrobenzoic acid (DTNB) by compounds containing sulfhydryl groups. Blood free sulfhydryl groups unrelated to proteins were derived almost only from GSH. The product of the described reaction is a compound of yellow color. Color density was measured at 412 nm. The calculations used the molar absorption coefficient, which, when attached to the mentioned wavelength, is equal to 13.6[mol^−1^ × l × cm^−1^]. The results were expressed in mmol/LRBC. The coefficient of variation for this method was 2.4%.

The activity of glutathione peroxidase (GPx) in erythrocytes was assayed by a two-stage Paglia and Valentine method [22]. In the first stage, GPx reacts with tert-butyl peroxide and reduced glutathione (GSH). The product of this reaction is glutathione disulfide (GSSG). The second stage involves the action of glutathione reductase (GR) reducing GSSG to GSH with the participation of NADPH+H+ as a regulator. NADPH oxidation results in a reduction in absorbance at a wavelength of 340 nm, which is measured spectrophotometrically.

cGPx activity was calculated based on the loss of the reduced form of coenzyme in time (test Wartburg). In the calculations, millimolar absorption coefficient for NADPH at 340 nm, equal to 6.22 [mmol^−1^ × l × cm^−1^], was used. The results were expressed in U/g Hb, where 1 *μ*mol oxidation of NADPH in one minute at *T* = 25°C was adopted as a unit of enzyme activity. The coefficient of variation for this method was 2.9%.

Determination of glutathione S-transferase (GST) activity in RBCs was performed according to the method of Habig and Jakob [23]. In this method, there is a decrease in absorbance (which is measured at a wavelength of 340 nm) due to the formation of a conjugate of glutathione (GSH) with 1-chloro-2,4-dinitrobenzene (CDNB). The decrease in absorbance is proportional to the glutathione S-transferase activity. GST activity assay was carried out in the presence of phosphate buffer and CDNB. The results were expressed in nmol/CDNB-GSH/mg Hb/min.

Superoxide dismutase (SOD-1) activity in RBCs was determined using the Misra and Fridovich method, which is based on the inhibition of adrenaline oxidation reaction by superoxide dismutase at pH 10.2 [24]. The increase in absorbance was measured at a wavelength of 480 nm. It is proportional to the increase in the concentration of oxidation products of adrenaline. The activity of SOD-1 was expressed in U/g Hb. The amount of enzyme which inhibits the oxidation of adrenaline 50% was adopted as a U unit. The coefficient of variation for this method is 6.3%.

The concentration of malondialdehyde (MDA) in the erythrocytes was determined by the Placer et al. method, which is based on the reaction of thiobarbituric acid and certain products of lipid peroxidation, mainly MDA, in an acidic environment and at elevated temperature [25]. This reaction produces a colored product, the color intensity of which was measured at a wavelength of 532 nm. In the calculations, the millimolar absorption coefficient of 156 [mmol^−1^ × l × cm^−1^] was used. The result was expressed in mmol/g Hb. The coefficient of variation for this method was 3.5%.

The concentration of nitric oxide was determined using the indirect method according to Marlett, determining the concentration of nitrate/nitrite in plasma. The method is based on the reaction between the nitrate anion and anion from N-(1-naphthyl)ethylenediamine, in the sulfanilic acid environment (Griess reaction) [26]. This reaction produced a colored complex whose absorbance is measured at a wavelength of 545 nm. It is directly proportional to the concentration of nitrates and nitrites in the studied sample. The result was expressed in *μ*ml/L.

Ceruloplasmin oxidase activity was determined using the method of Ravin [27]. The principle of the method is based on oxidation of substrate p-phenyldiamine (PPD) by ceruloplasmin at a final purple-colored product. Absorbance measurement was made at a wavelength of 530 nm. This product is so called “the principle of Bandrowski” (product formed from three molecules of the substrate). Results were expressed in international units.

### 2.3. Statistical Analysis

To evaluate the significance of changes after intervention, paired Student's t-test was performed. The Shapiro–Wilk test was performed to evaluate the normality of the variables. The results were shown as mean and standard deviation (SD). Additionally, ±95% confidence intervals (CIs) were calculated for the changes after intervention. The effect size of the observed changes was estimated using Cohen's d statistics, were values below 0.1, 0.3, 0.5, 0.7, and 0.9 indicate trivial, small, moderate, large, and very large effect, respectively [28]. Statistical analysis was performed using IBM SPSS Statistics v. 12. The difference was statistically significant at p < 0.05. The minimal sample size of 19 participants was estimated using the G∗Power software ver. 3.1.9.4 (Franz Faul et al., Universität Kiel, Germany) for large effect size and power of 0.80. The additional ten participants were enrolled in case of any dropouts which is shown in Figure 1.

As a result of the therapy, no changes in the levels/concentration of the measured parameters of the oxidative stress were observed in HT, GSH, NO_2-_/NO_3-_, and CP. Contrary, it was shown that after massage, there was a significant decrease about 8% and 13% in the level/concentration of GPx_RBC_ and MDA, respectively as shown in Table 1. The study demonstrated also a significant increase of 16% and 7% in the level/concentration of GPxp and SOD-1, after massage, respectively as show in (Figure 2).

## 3. Discussion

The internal balance of the organism is perceived systemically, but also at the cellular and subcellular level. Lifestyle, leisure activities, improper diet, and application of stimulants may provoke generation of various oxygen forms in the organism. On the other hand, every prohealth initiative such as physical activity, optimal diet, and physiotherapy (including massage) may decrease the risk of free radical-related diseases. Systemic and local antioxidant systems depend also on age—they are less efficient in children and adolescents than in middle-aged people, which indicates also age-related immaturity of antioxidant mechanisms [29]. Our results confirmed the hypothesis concerning influence of classical massage on selected parameters of oxidative stress, including GPx_RBC_, GPxp, SOD-1, and MDA.

Integrated and effective human defense system is needed to control the production of free radicals as well as counteract their biological consequences. Extensive production of ROS may be limited/balanced. Aforementioned defense system should consist of both enzymatic and nonenzymatic mechanisms that dispose ROS.

Physiotherapy may play a significant role in this process [30]. Current evidence concerning influence of classical massage on oxidative stress is limited. Study by Karabulut et al. [19] showed that regular physical activities combined with postexercise massage increase SOD-1 activity and do not change adenosine deaminase (ADA). Such outcome supports the assumption that regular physical activity and massage has favorable health effects. Our results are consistent with aforementioned results in SOD-1. However, it should be noted that Karabulut et al. [19] investigated effects of physical exercise alone and in combination with massage, but not massage alone. Moreover, the final outcome was similar regardless of the massage intervention. Analogous results are presented by Heydari et al. who showed that the use of various forms of massage during recovery and rest after exhausting physical exertion may also influence SOD level. [13]

Study by Amano et al. showed that overall health care program, including body massage (cupping and vibration), may significantly improve health status (including oxidative stress) of the preobese or mildly obese middle-aged women. It is difficult to point to the key factor that had impact on health of the examined women. The influence of massage alone was not investigated in the aforementioned findings, yet it may play an important role in comprehensive approach [31].

Presented outcome may support evidence that classical massage may prove helpful in neutralizing radical superoxide by enzymatic defense system [29], which is also confirmed in the given study by the fact that an increased activity of GPx was observed after massage, as compared to the values before the massage. This result is consistent with the results presented by Heydari et al. [13]. Another important parameter of oxidative stress is GST, taking part i.a. in regulation of GPx [32]. Our studies show lack of differences in the GST activity before/after the massage. Similar outcome is observed by Ciechomski et al. [33] who assess GPx and GSH in patients relaxing after training (passively or undergoing massage). The effect of the damages caused by oxidative stress may be also measured indirectly using MDA [34]. MDA concentration increases with extensive production of ROS in the organism [35]. Our study showed a decrease in MDA level after massage compared to the value before the massage. Similar results were presented by Heydari et al. and Karabulut et al. [13, 19]. NOx also play an important role as an element of antioxidant barrier of the organism [36, 37]. Our study has failed to show a significant impact of the massage. The outcome is similar to the one showed by Karabulut et al. [19]. Another important parameter of oxidative stress is CP [38]. We have not observed significant differences in CP level before/after massage.

The mechanism of the observed reaction may be due to the microdamage of the muscles after the massage. Activation of monocytes, increasing the expression of inflammatory cytokines leads to the activation of endothelial leukocyte adhesion molecules P-selectin and E-selectin. Neutrophils intensify the breakdown of tissue, leading to the release of free radicals in the environment and, consequently, a change in the studied parameters [39].

Main limitations of our study included a relatively small group of volunteers and no placebo group; thus, we regard our study as preliminary. Only immediate results of the massage therapy on selected biochemical parameters of the oxidative stress were assessed during the study. Long-term results will be assessed during further studies. Moreover, we assessed only the influence of the single session of the therapeutic massage. Cumulative effect of the subsequent massage therapy sessions may be stronger or longer-lasting.

Further studies require randomized controlled trials on bigger number of volunteers, as well as taking into consideration such factors as sex, age, previous lifestyle, diet, and body mass index. Such detailed approach would allow assessment of possible prognostic signs and provide scenarios for prohealth prevention in various groups of patients.

Other parameters of oxidative stress may be used in treating disease-related complications as well as in the interdisciplinary treatment. Intensity of the massage (and associated physical exercises), its duration, and used techniques may also influence development of the oxidative stress and its long-term consequences. The ultimate goal is optimization of classical massage in prevention and treatment of oxidative stress in both healthy and ill people, including elderly patients [40–43].

## Figures and Tables

**Figure 1:** Patient flow diagram.

**Figure 2:** Percentage of changes in mean values of selected measured parameters of oxidative stress before and after classical massage.

**Table 1:** Mean values of activity or concentration of the selected parameters of oxidative stress before and after classical massage.

Parameter	Before (n = 29)		After (n = 29)		±95% CI of change	p value	Cohen's d
	Mean	SD	Mean	SD			
HT	43.845	3.303	43.862	3.359	0.112; -0.078	0.713	0.005
GSH (mmol)	2.441	0.258	2.441	0.261	0.020; -0.019	0.971	0.001
GPxp (U)	237.797	38.932	282.010	58.625	60.443; 27.985	0.001	0.888
GPx_RBC_ (U)	18.431	2.358	16.945	2.323	-0.922; -2.050	0.001	-0.635
GST (nmol)	3.007	0.674	2.910	0.627	0.067; -0.260	0.236	-0.149
SOD-1 (U)	2648.620	334.480	2844.140	374.743	258.960; 132.074	0.001	0.550
MDA (mmol)	0.291	0.029196	0.253	0.514	-0.021; -0.053	0.001	-0.102
NO_2-_/NO_3_ (*μ*mol/L)	3.117	3.267	3.240	3.139	0.801; -0.555	0.713	0.038
CP (IU)	1141.676	391.677	1148.334	375.960	44.287; -30.970	0.720	0.017

HT: hematocrit; GSH: glutathione; GPxp: glutathione peroxidase (plasma); GPx_RBC_: glutathione peroxidase (red blood cells); GST: glutathione S-transferase; SOD-1: superoxide dismutase; MDA: malondialdehyde; NO_2_/NO_3_: nitrate/nitrite; CP: ceruloplasmin oxidase.

## Data Availability

The biochemistry data used to support the findings of this study are included within the article.

## Abbreviations

CAT: Catalase
CP: Oxidase ceruloplasmin
GPx: Glutathione peroxidase
GPxp: Glutathione peroxidase (plasma)
GPx_RBC_: Glutathione peroxidase (red blood cells)
GR: Glutathione reductase
GSH: Glutathione
GST: Glutathione S-transferase
H_2_O_2_: Hydrogen peroxide
HT: Hematocrit
MDA: Malondialdehyde
NO_2_: Nitrate
NO_3_: Nitrite
O_2_: Singlet oxygen
O_2-_: Superoxide anion
O_3_: Ozone
OH: Hydroxyl radical
RO: Alkoxy radical
ROO: Radical peroxide
ROS: Reactive oxygen species
SD: Standard deviation
SOD-1: Superoxide dismutase.
